# PCAT19 Regulates the Proliferation and Apoptosis of Lung Cancer Cells by Inhibiting miR-25-3p via Targeting the MAP2K4 Signal Axis

**DOI:** 10.1155/2022/2442094

**Published:** 2022-05-16

**Authors:** Bing Wang, Shengrong Yang, Yang Jia, Jianru Yang, Kun Du, Yujie Luo, Yunhe Li, Zhenghong Wang, Yi Liu, Bing Zhu

**Affiliations:** ^1^Department of Thoracic and Cardiovascular Surgery, The Second Affiliated Hospital of Chongqing Medical University, No. 76, Linjiang Road, Yuzhong District, Chongqing 400010, China; ^2^Department of Plastic Surgery, The Second Hospital of Hebei Medical University, No. 215, West Heping Road, Shijiazhuang, Hebei Province 050000, China; ^3^Department of Obstetrics and Gynecology, The Second Affiliated Hospital of Chongqing Medical University, No. 76, Linjiang Road, Yuzhong District, Chongqing 400010, China

## Abstract

Both PCAT19 and miR-25-3p have been reported in lung cancer studies, but whether there is a correlation between the two and whether they jointly regulate the progress of lung cancer have not been reported yet. Therefore, this study carried out a further in-depth research. The expression of PCAT19 was detected in lung cancer (LC) tissues and cells by quantitative real-time polymerase chain reaction (qRT-PCR). The effect of PCAT19 on tumor growth was detected in a tumor-bearing model of nude mice. PCAT19-transfected cells were treated with Honokiol and anisomycin. The effects of PCAT19 on proliferation, apoptosis, and cycle of LC cells were investigated by biomolecule experiments. The effects of PCAT19 on the expressions of mitogen-activated protein kinase- (MAPK-) related proteins were evaluated by western blotting. The expression of PCAT19 was decreased in LC tissues and related to patient survival, tumor size, and pathology. In addition, upregulation of PCAT19 hindered LC cell proliferation, miR-25-3p expression, and the activation of extracellular regulated protein kinases (ERK) 1/2, p38, and c-Jun N-terminal kinase (JNK), while facilitating LC cell apoptosis. Furthermore, upregulation of PCAT19 reversed the effects of Honokiol and anisomycin on promoting cell proliferation and inhibiting cell apoptosis. Collectively, our findings show that upregulated PCAT19 suppresses proliferation yet promotes the apoptosis of LC cells through modulating the miR-25-3p/MAP2K4 signaling axis.

## 1. Introduction

According to the latest statistics, there are approximately 235,760 cases of lung and bronchial cancer being diagnosed and 131,880 deaths in 2021 (Siegel et al. [1]). Lung cancer (LC) is a frequently diagnosed malignant tumor, with the highest morbidity and mortality worldwide (Torre et al. [2], Goubran et al. [3]). At present, the treatment of early lung cancer is often based on comprehensive treatments such as surgery, radiotherapy, and chemotherapy and Chinese medicine (Wangari-Talbot and Hopper-Borge [4]). Although advances have been made in the treatment of lung cancer, the 5-year survival rate of LC patients has not been improved greatly, and the mortality rate of LC remains the highest as compared with that of other cancer deaths (Baghdadi et al. [5]). Though the etiology of LC has not yet been fully clarified, there are data indicating that the occurrence of is closely related to assorted factors such as living habits, family inheritance, and endocrine disorders (Avci et al. [6], Granger et al. [7], Dreher et al. [8]). Molecular biology studies have revealed that the occurrence of LC is caused by abnormal proliferation, differentiation, and apoptosis of cells, and these abnormal biological behaviors are associated with abnormal molecular expression, activation, and mutation *in vivo* (Zhao et al. [9], Jiang et al. [10]). Thus, comprehensive discovery and further exploration on the functions and regulatory mechanisms of these related molecules could help us to understand the molecular mechanism of LC and provide a more effective target for LC treatment.

It is widely recognized that long noncoding RNAs (lncRNAs) make profound impacts on the regulation of gene expressions, and their abnormal expressions are associated with various diseases. As previously reported, lncRNAs are also involved in the occurrence and development of tumors through acting as protooncogenes or tumor suppressor genes (Engreitz et al. [11], Liu and Zhao [12], Wang et al. [13]). Several studies have found that lncRNA PCAT19 plays a carcinogenic role in prostate cancer and laryngeal cancer (Hua et al. [14], Xu, Guo, and Zhang [15]), but its role in LC is less reported. Therefore, the current study was aimed at fathoming out the mechanism of action of PCAT19 in LC.

A mutual regulatory relationship has been corroborated between lncRNA and microRNA (miRNA) (Chen et al. [16], Wang, Jia, et al. [17]), where lncRNAs can interact with miRNA through acting as a competitive endogenous RNA and participate in the regulation of target gene expressions (Yoon, Abdelmohsen, and Gorospe [18], Hao et al. [19]). miRNAs produce their biological effects via an RNA-induced silencing complex to regulate lncRNA. Moreover, miRNA and lncRNA both participate in the occurrence of various diseases (He et al. [20]). A previous study has indicated that miR-25-3p is highly expressed in LC tissues (Giordano et al. [21]). However, whether there is a targeting relationship between PCAT19 and miR-25-3p and whether such a relationship participates in the development of LC remain to be further determined. Thus, this study was dedicated to probing into the potential mechanisms of PCAT19 and miR-25-3p in LC. In addition to the fact that activated mitogen-activated protein kinase (MAPK) is involved in physiological processes such as cell proliferation, differentiation, migration, apoptosis, and stress response, the present studies also found that MAPK is implicated in the occurrence and development of diversified tumors, including those in LC (Hu et al. [22], Wang, Jia, et al. [17]), and that activation of protein kinase B (AKT) and extracellular regulated protein kinase (ERK-) MAPK signaling pathways could mediate the downstream effects of miR-25-3p, which in turn promotes tumor cell proliferation (Chen et al. [23]). In the current study, LC cells were subjected to the treatment with MAPK signaling pathway-associated agonists for further investigating whether PCAT19 regulated the progression of LC through modulating the MAPK signaling pathway.

## 2. Material and Methods

### 2.1. Biological Information Analysis

Gene Expression Profiling Interactive Analysis (GEPIA) was applied to predict the expression of PCAT19 in LC. The binding sites between PCAT19 and miR-25-3p were predicted by using LncBase Predicted v.2, and those between miR-25-3p and MAP2K4 were analyzed by using TargetScan 7.2.

### 2.2. Clinical Specimens

LC tissue and adjacent tissue samples were obtained from 74 cases of LC patients who attended the Second Affiliated Hospital of Chongqing Medical University for treatment from January 2018 to May 2019. Patients with lung cancer included in the study had not undergone any treatment before. Their tissue samples were kept in liquid nitrogen and maintained at -80°C. All subjects signed the written informed consent, and the current study was approved by the Ethics Committees of the Second Affiliated Hospital of Chongqing Medical University.

### 2.3. Dual-Luciferase Reporter Assay

The PCAT19 sequence containing miR-25-3p binding sites was inserted into the pmirGLO dual-luciferase vector (Promega, USA) to generate wild-type (WT) pmirGLO-PCAT19. The mutant (Mut) PCAT19 sequence in the miR-25-3p binding site was synthesized by using a Site-Directed Mutagenesis Kit (F542, Thermo Fisher Scientific, USA) and then inserted into the pmirGLO dual-luciferase vector to generate Mut pmirGLO-PCAT19. Similarly, the 3′ UTR of MAP2K4 containing the predicted miR-25-3p-binding sites or Mut sites was inserted into the pmirGLO dual-luciferase vector as pmirGLO-MAP2K4-3′UTR-WT and pmirGLO-MAP2K4-3′UTR-Mut, respectively. The pmirGLO vector containing the WT or Mut PCAT19 sequence and WT or Mut MAP2K4 3′ UTR was cotransfected with the miR-25-3p mimic into A549 and SK-MES-1 cells by using Lipofectamine2000 (Invitrogen, USA), respectively. After incubation for 48 h, the relative luciferase activity of the cells was measured by the Dual-Luciferase Reporter Assay protocol (Promega, Madison, WI).

### 2.4. Cell Culture and Transfection

BEAS-2B was used as the human normal lung epithelial cell line, while A549, H1299, and SK-MES-1 were LC cell lines. The cells were purchased from the Cell Bank of the Chinese Academy of Sciences (Shanghai, China) and cultured in RPMI-1640 (Gibco, USA) containing 10% fetal bovine serum (FBS, Gemini Bio-Products, Sacramento, CA) at 37°C with 5% CO_2_. The cells at the logarithmic growth stage were selected for experiments.

In the three LC cell lines, as PCAT19 was lowly expressed in A549 cells but highly expressed in SK-MES-1, A549 and SK-MES-1 cells were singled out for the following experiments. To explore the effects of PCAT19 on the A549 and SK-MES-1 cells, the cells were divided into a negative control (NC) group, PCAT19 group, siNC group, siPCAT19 group, Honokiol group, anisomycin group, PCAT19+Honokiol group, and PCAT19+anisomycin group. A549 and SK-MES-1 cells were treated with 10 *μ*M Honokiol ERK agonist (98% purity, Nacalai Tesque, Japan) and 0.1 *μ*M anisomycin p38 and c-Jun N-terminal kinase (JNK) agonist (98% purity, Nacalai Tesque, Japan).

The cells were digested, thoroughly mixed, seeded into the 6-well plates at a concentration of 1 × 10^6^ cells/mL, and then evenly distributed in an orifice plate to reach 80-90% confluence. 20 pmol recombinant adenovirus of the pLJM1 vector (60908-4538, TIANDZ, Beijing, China) with PCAT19, siPCAT19, and siNC (Shanghai GenePharma Co., Ltd., China) was separately dissolved in gradient in 180 *μ*L Dulbecco's modified Eagle medium (DMEM, HyClone, USA). The cells transfected with the pLJM1 empty vector were applied as the NC group. Next, the cell transfection was performed by using Lipofectamine2000 according to the manufacturer's instructions. Transfected cells were cultured in the 6-well plates at 37°C with 5% CO_2_. The medium was changed 2 h after the transfection, and the cells were collected after culture for 72 h.

### 2.5. Quantitative Real-Time Polymerase Chain Reaction (qRT-PCR)

Total RNA was extracted from the cells using the TRIzol reagent (15596018, Thermo Fisher Scientific, USA), and the concentration of the RNA was detected by using Nanodrop (FSC-6539918, eGeneralMedical.com, USA) and diluted to 500 ng/*μ*L. For miRNAs, NCode VILO miRNA cDNA Synthesis and EXPRESS SYBR GreenER miRNA qRT-PCR Kits (Life Technologies) were applied for detecting the expression levels. For mRNAs, total RNA (1 *μ*g) was converted into cDNAs using a Superscript II first-strand cDNA synthesis system (Invitrogen, USA). The mRNA expression levels were determined by SYBR-Green PCR Master Mix (Thermo Fisher Scientific, USA) in the 7500 Real-Time PCR system (Thermo Fisher Scientific, USA). Conditions of the PCR cycle were set as follows: pretreatment at 95°C for 30 s, followed by 60°C for 30 s and 60°C for 30 s for 45 cycles. The 2^−ΔΔCT^ method was used to determine the expression levels of RT-PCR products (Livak and Schmittgen [24]). All primer sequences used are listed in Table 1.

### 2.6. Cell Viability Detection

The cells were inoculated into the 96-well plate at a density of 5 × 10^3^ cells/well and cultured with 10% fetal bovine serum (FBS, Gibco, USA) at 37°C with 5% CO_2_. Next, 20 *μ*L methylthiazolyldiphenyl-tetrazolium bromide (MTT) solution (C0009, Beyotime Biotechnology, China) was added into each well, and the cells were cultured for 4 h. Then, 150 *μ*L 0.5% DMSO was added into each well, and the plate was shaken gently for 10 min to fully dissolve the purple crystals. The absorbance at 492 nm was read using a microplate reader (E0225, Beyotime Biotechnology, China). All the experiments were performed in triplicate, and the average value was calculated.

### 2.7. Colony Formation Assay

The cells were transfected, digested, counted, and then cultured in 12-well plates at a density of 100 cells per well at 37°C in 5% CO_2_ for 2 weeks. The conditioned medium was changed every 3 days to observe clone formation. The culture was terminated when the cloned cells were observed within 50-150 fields. Then, the medium was discarded, and the cells were rinsed twice in Dulbecco's Phosphate-Buffered Saline (DPBS, D8662, Sigma-Aldrich, USA). Later, the cells were fixed with 1 mL methanol (34860, Sigma-Aldrich, USA) for 15 min and stained with 1 mL Giemsa staining solution (G5637, Sigma, USA) for 30 min. Ultimately, the colony formation rate was calculated using the following formula: colony formation rate = (number of colonies/number of seeded cells) × 100%. Each treatment was carried out in triplicate.

### 2.8. Cell Apoptosis

The cells were resuspended by RPMI-1640 and centrifuged at 1000 × *g* for 5 min at 4°C. Subsequently, the supernatant was discarded, and the cells were resuspended in 1× Annexin Binding Buffer consisting of 5 *μ*L fluorescein isothiocyanate- (FITC-) Annexin V and 1 *μ*L 100 *μ*g/mL propidium iodide (PI) (85-BMS500PI, MULTI SCIENCES, Hangzhou, China), and the cell suspension was then added with 300 *μ*L 1× Annexin Binding Buffer and subsequently held at room temperature for 15 min. Finally, the stained cells were analyzed by flow cytometry.

### 2.9. Cell Cycle

The cells at the log phase of growth (1 × 10^6^/mL) were collected, trypsinized, washed with PBS three times, and fixed with 3 mL 70% iced ethanol at 4°C for 48 h. After that, the fixed cells were stained with 400 *μ*L 50 *μ*g/mL PI solution and analyzed with a flow cytometer (version 10.0, FlowJo, FACSCalibur™, BD, Franklin Lakes, NJ, USA).

### 2.10. Western Blotting

The total proteins of cells were lysed by RIPA Lysis and Extraction Buffer (89901, Thermo Fisher Scientific, USA) and centrifuged at 1000 × *g* for 5 min at 4°C. The protein concentration was determined by using the BCA protein kit (QPBCA, Sigma-Aldrich, USA). Next, the proteins were separated on 15% dodecyl sulfate sodium salt-polyacrylamide gels (SDS-PAGE) and then transferred to polyvinylidene fluoride membranes (EMD Millipore, USA). Next, the membranes were blocked with 5% nonfat milk at room temperature for 1 h, and the blots were then incubated with the primary antibodies against p-ERK1/2 (rabbit, 1 : 1000, #9101, Cell Signaling Technology (CST)), ERK1/2 (rabbit, 1 : 1000, #4695, CST), anti-p-p38 (rabbit, 1 : 1000, #4631, CST), p38 (rabbit, 1 : 1000, #9212, CST), p-JNK (rabbit, 1 : 1000, #4668, CST), JNK (rabbit, 1 : 1000, #9252, CST), and GAPDH (mouse, 1 : 10000, #5174, CST) at 4°C overnight. The membranes were washed with PBS three times and then incubated with secondary antibody goat anti-mouse or goat anti-rabbit IgG (H+L) (Proteintech, USA) for 2 h, respectively, and then washed with TBST for three times. Afterwards, the membranes were developed, and the protein bands were detected using the ECL kit (MAB5350, Sigma-Aldrich, USA) and scanned with a supersensitive multifunctional imager (ImageJ, version 4.7, Amersham Imager 600, GE).

### 2.11. Establishment of the Tumor-Bearing Model in Nude Mice

Sixteen athymic nude mice (6 weeks old, 20 ± 2 g, male) were purchased from Shanghai Lab, Animal Research Center (license no. SCK (Shanghai) 2008-0016, China) and housed under specific disease-free (SPF) conditions. Ethical and legal approval of animals was obtained from Zhengzhou University. All experiments were performed following institutional and national guidelines and regulations of Zhejiang University. The mice were raised under the temperature of 18-25°C and the humidity of 40-70%. Animals were lived in the day-night cycle of 12 to 12 h with the supplement of regular feed and fertilized water. The mice were divided into two groups, namely, NC group (*n* = 8) and PCAT19 group (*n* = 8). 200 *μ*L 1× PBS was used to resuspend the A549 cells transfected with PCAT19 or NC (1 × 10^5^/mL). In the NC group, A549 cells transfected with NC were injected into the right flank of each mouse (weighing 25 g). In the PCAT19 group, A549 cells transfected with PCAT19 were injected into the right flank of each mouse (weighing 25 g).

After being fed for 27 days, all the mice were sacrificed and their tumors were weighed. During the experiment, length and width of the mouse tumor were measured by using Vernier calipers every 3 days, and tumor volumes were measured according to the formula as follows: the *V* (mm^3^) = largest diameter × perpendicular diameter^2^/2. Tumor tissues of the mice from the two groups were extracted for immunohistochemistry and terminal deoxynucleotidyl transferase (TdT) dUTP nick-end labeling (TUNEL) assay.

### 2.12. Immunohistochemical Staining

The subcutaneous tumor tissues of nude mice were fixed with formaldehyde (SF877503, Sinopharm Chemical Reagent Beijing Co., Ltd., China), dehydrated with gradient alcohol (80%, 90%, 95%, and 100%), and transparentized with xylene (10023418, Sinopharm Chemical Reagent Beijing Co., Ltd., China). Next, the tissues were wax-immersed, paraffin-embedded, and finally sectioned into tissue slices. Then, the tissue slices were dewaxed with xylene, dephenylated with ethanol at the concentrations of 100%, 95%, 80%, and 70% for 2 min, and washed with PBS twice. After that, 30 mL EDTA antigen repair buffer (P0086, Beyotime Biotechnology, China) was diluted with 1,500 mL distilled water and then boiled in a microwave box. Next, the tissue slices were completely immersed in the buffer to repair antigen, heated for 10 min, naturally cooled, and rinsed in PBS for three times. Following these, each tissue slices were added with 3 drops of 3% H_2_O_2_, incubated under light at room temperature for 15 min to eliminate the activity of endogenous peroxidase, and then washed with PBS three times. Subsequently, the tissue slices were incubated with a primary antibody (anti-Ki-67, ab15580, Abcam, USA) at 4°C overnight and washed with PBS for three times. Afterwards, the tissue slices were ulteriorly cultivated with a secondary antibody at 37°C for 30 min and rinsed with PBS again for three times, followed by being stained with the DAB developing kit (P0202, Beyotime Biotechnology, China) and washed with distilled water for 1 min. Later, the cells were stained with hematoxylin for 1 min, washed under tap water for 30 min, and then sealed with gum. Eventually, the red and granulated cells were observed under an optical microscope (BX40, Olympus, Japan).

### 2.13. TUNEL Assay

Apoptosis was detected by using the TUNEL kit (Promega, USA). In brief, the tumor tissue samples were embedded with paraffin, sectioned (4 *μ*m), and digested with protease K for 30 min. Next, the tissue sections were incubated with TUNEL reaction fluid at 37°C for 1 h. Then, the streptavidin-HRP working solution (SNN1004, Thermo Fisher Scientific) was added to further incubate the sections at room temperature for 30 min. After that, the sections were stained with DAB chromogen, counterstained with hematoxylin, and dehydrated with ethanol at the concentrations of 70%, 80%, 90%, and 95%, respectively. Finally, the sections were observed under an optical microscope.

### 2.14. Statistical Analysis

Prism 6 (version 6.01, GraphPad Software, Inc., San Diego, CA, USA) was used for data analysis. The results were presented as mean ± standard deviation (SD) of at least 3 independent experiments. Student's *t*-test was performed to compare the differences in the mean between the continuous variables, while those among multiple groups were analyzed by one-way analysis of variance (ANOVA), followed by the Bonferroni post hoc test. The Kaplan-Meier plotter was employed to predict the relationship between PCAT19 and LC survival. The Spearman correlation was used to analyze the relationships among PCAT19, miR-25-3p, and MAP2K4. *P* < 0.05 was considered to be statistically significant.

## 3. Results

### 3.1. PCAT19 Was Lowly Expressed in LC Tissues and Cells

The GEPIA website was used to analyze the expression of PCAT19 in various cancers, and the results showed that PCAT19 appeared to have a low expression in 11 types of cancer (including breast invasive carcinoma (BRCA), cervical squamous cell carcinoma and endocervical adenocarcinoma (CESC), kidney chromophobe (KICH), kidney renal papillary cell carcinoma (KIRP), lung adenocarcinoma (LUAD), lung squamous cell carcinoma (LUSC), ovarian serous cystadenocarcinoma (OV), thyroid carcinoma (THCA), skin cutaneous melanoma (SKCM), uterine corpus endometrial carcinoma (UCEC), and uterine carcinosarcoma (UCS)), especially in LUAD and LUSC (Figure 1(a)). Besides, PCAT19 presented a low expression in LUAD and LUSC tissues compared with paracancer tissues (ANT) (*P* < 0.001, Figure 1(b)). Moreover, the relationship between PCAT19 and lung cancer survival was predicted by using the Kaplan-Meier plotter, and the result uncovered that LC patients with a high expression of PCAT19 had a higher survival rate (*P* < 0.001, Figure 1(c)).

### 3.2. Relationship between PCAT19 Expression Level and Clinical Characteristics of LC Patients

qRT-PCR was performed to detect the expression of PCAT19 in cancer tissues and ANT collected from 74 LC patients, and the results exhibited that PCAT19 was conspicuously downregulated in tissues of LC patients (*P* < 0.001, Figure 2(a)), with the mean PCAT19 expression level being 4 ± 1.2 (Figure 2(B)). In this research, the LC patients with PCAT19 expression lower than the average level were defined as having low expression of PCAT19 (*n* = 34), while those with the expression higher than the average level were identified as having high expression of PCAT19 (*n* = 40). In addition, the relationship between PCAT19 and clinical characteristics of the patients was analyzed. As illustrated in Table 2, we found that PCAT19 expression was related to tumor size and pathology (*P* < 0.05), but not associated with age (*P* = 0.859), gender (*P* = 0.719), clinical stage (*P* = 0.423), or lymph node metastasis (*P* = 0.370). Furthermore, the expression of PCAT19 in the human normal lung epithelial cell line (BEAS-2B) and LC cell lines (A549, H1299, and SK-MES-1) was also detected by qRT-PCR, and the result mirrored that PCAT19 level was downregulated in LC cell lines (*P* < 0.001, Figure 2(c)).

### 3.3. Upregulated PCAT19 Inhibited LC Cell Proliferation

PCAT19 and siPCAT19 vectors were transfected into A549 and SK-MES-1 cells to further investigate the effect of PCAT19 on proliferation of LC cells. As depicted in Figures 3(a) and 3(b), PCAT19 and siPCAT19 vectors were successfully transfected into LC cells. Furthermore, the MTT assay was performed to detect the viabilities of A549 and SK-MES-1 cells transfected with PCAT19 and siPCAT19 vectors at 24 h, 48 h, and 72 h, and the results revealed that overexpression of PCAT19 inhibited cell viability, whereas PCAT19 silencing increased cell viability at 48 h and 72 h (*P* < 0.05, Figures 3(c) and 3(d)). Moreover, the colony formation assay was performed to observe the proliferation of PCAT19- and siPCAT19-transfected LC cells, and the data demonstrated that overexpression of PCAT19 inhibited the colony numbers of A549 and SK-MES-1 cells, while PCAT19 silencing enhanced the colony numbers of A549 and SK-MES-1 cells (*P* < 0.001, Figures 3(e) and 3(f)).

### 3.4. Upregulated PCAT19 Promoted LC Cell Apoptosis

The effects of PCAT19 on apoptosis of A549 and SK-MES-1 cells were evaluated by flow cytometry. The results unraveled that overexpression of PCAT19 promoted apoptosis, while PCAT19 silencing inhibited apoptosis (*P* < 0.001, Figures 3(g) and 3(h)). Moreover, overexpressed PCAT19 displayed an increase in G1 and a decrease in the S phase, and A549 and SK-MES-1 cells were blocked in the G1 phase. At the same time, PCAT19 silencing presented a decrease in the G1 phase and an increase in the S phase, and the cells transformed into the G-S phase (*P* < 0.05, Figures 3(i) and 3(j)). Furthermore, we explored the effects of PTCA19 on the LC tumor by establishing a tumor-bearing model in nude mice for *in vivo* experiments and discovered that the volume and weight of the tumor were reduced dramatically in the PCAT19 treatment group compared with the NC group (*P* < 0.001, Figures 4(a)–4(c)). Furthermore, immunohistochemistry exhibited that the expression of Ki-67 was reduced, but the cell apoptosis was increased in the PCAT19 group, as compared with the NC group (*P* < 0.001, Figure 4(d)).

### 3.5. PCAT19 Regulated the miR-25-3p/MAP2K4 Signaling Axis

In the A549 and SK-MES-1 cells, PCAT19 was highly expressed in the cytoplasm yet lowly expressed in the nucleus (*P* < 0.001, Figures 5(a) and 5(b)). LncBase Predicted v.2 predicted that there were binding sites between PCAT19 and miR-25-3p (Figure 5(c)). To further confirm this prediction, we constructed two pmirGLO dual-luciferase reporter vectors, namely, PCAT19-3′-UTR wt and PCAT19-3′-UTR mut (hereafter PCAT19-WT and PCAT19-Mut), then separately cotransfected them with the miR-25-3p mimic into A549 and SK-MES-1 cells, and observed that the luciferase activity of PCAT19-WT was obviously suppressed (*P* < 0.001, Figures 5(d) and 5(e)), while no prominent changes were found on the luciferase activity of PCAT19-Mut. Furthermore, TargetScan 7.2 predicted that the MAP2K4 had complementary base pairing with miR-25-3p (Figure 5(f)). To further confirm that, two pmirGLO-dual-luciferase reporter vectors, MAP2K4-3′-UTR wt and MAP2K4-3′-UTR mut (hereafter MAP2K4-WT and MAP2K4-MUT), were constructed. Subsequently, these two vectors were cotransfected with the miR-25-3p mimic into A549 and SK-MES-1 cells, respectively. The results uncovered that the luciferase activity of cells cotransfected with MAP2K4-WT and miR-25-3p mimic was remarkably suppressed, and that of cells cotransfected with MAP2K4-Mut and miR-25-3p mimic was not signally altered, signifying that MAP2K4 was the target gene of miR-25-3p (*P* < 0.001, Figures 5(g) and 5(h)).

### 3.6. Expression and Correlation Analysis of miR-25-3p and MAP2K4 in LC Tissues

The expressions of miR-25-3p and MAP2K4 in LC tissues and ANT of 74 LC patients were detected by qRT-PCR, and the data demonstrated that miR-25-3p level was upregulated and MAP2K4 level was downregulated in the LC tissues (*P* < 0.001, Figures 6(a) and 6(b)). The data from the Spearman correlation analysis demonstrated that PCAT19 was negatively correlated with miR-25-3p (*P* < 0.001, Figure 6(c)), miR-25-3p was negatively correlated with MAP2K4 (*P* < 0.001, Figure 6(d)), and PCAT19 was positively correlated with MAP2K4 (*P* < 0.001, Figure 6(e)).

### 3.7. Upregulated PCAT19 Inhibited the Activation of the MAPK Signaling Pathway

We detected the effects of PCAT19 on the MAPK signaling pathway by western blotting, and the results unraveled that the expressions of MAPK signaling pathway-related proteins (p-ERK1/2, p-p38, and p-JNK) were markedly inhibited in A549 and SK-MES-1 cells transfected with the PCAT19 overexpression vector (*P* < 0.001, Figures 7(a)–7(d)), while PCAT19 silencing augmented the expressions of MAPK signaling pathway-related proteins (p-ERK1/2, p-p38, and p-JNK) in A549 and SK-MES-1 cells (*P* < 0.001, Figures 7(a)–7(d)). In addition, the ratios of MAPK signaling pathway-related proteins were calculated in A549 and SK-MES-1 cells, and we found that the ratios of p-ERK1/2/ERK1/2, p-p38/p38, and p-JNK/JNK were visibly reduced in A549 and SK-MES-1 cells transfected with the overexpressed PCAT19 vector (*P* < 0.001, Figures 7(e) and 7(f)), while the ratios of p-ERK1/2/ERK1/2, p-p38/p38, and p-JNK/JNK were prominently increased in the A549 and SK-MES-1 cells transfected with the siPCAT19 (*P* < 0.001, Figures 7(e) and 7(f)).

### 3.8. PCAT19 Regulated LC Cell Growth via Inhibiting the MAPK Signaling Pathway

After A549 and SK-MES-1 cells were treated with 10 *μ*M Honokiol (ERK agonist) or 0.1 *μ*M anisomycin (p38 and JNK agonist) and transfected with the PCAT19 overexpression vector, the viability of A549 and SK-MES-1 cells was detected by the MTT assay, and the results revealed that the cell viability in the PCAT19 group was lower than that in the NC group, the cell viability of Honokiol and anisomycin groups was higher than that of the NC group, and the cell viability of PCAT19+Honokiol and PCAT19+anisomycin groups was lower than that of Honokiol and anisomycin groups, respectively (*P* < 0.001, Figures 8(a) and 8(b)). In addition, the colony numbers in PCAT19+Honokiol and PCAT19+anisomycin groups were lower than those in Honokiol and anisomycin groups, respectively (*P* < 0.001, Figures 8(c) and 8(d)). Furthermore, the results of flow cytometry showed that apoptosis in PCAT19+Honokiol and PCAT19+anisomycin groups was overtly higher than that in Honokiol and anisomycin groups, respectively (*P* < 0.001, Figures 8(e) and 8(f)).

## 4. Discussion

The pathogenesis of LC has been affirmed to be closely related to malignant proliferation and differentiation disorders of cells (Hu et al. [25]). Therefore, investigating the molecular mechanism of LC is of great significance for understanding the occurrence and development of LC, so as to make effective therapeutic regimens for LC patients. Increasing studies have corroborated that the abnormal expressions of lncRNAs are involved in the occurrence and development of tumor cells, and much attention has been focused on the modulating the expressions of lncRNA-related genes to reverse the growth of tumor cells (Engreitz et al. [11], Liu and Zhao [12]).

Studies conducted on PCAT19 in prostate cancer and laryngeal cancer (Gao, Xia, et al. [26], Xu, Guo, and Zhang [15]) demonstrated that aggressiveness of prostate cancer is positively associated with increased expression of PCAT19 Gao, Xia, et al. [26], and upregulation of PCAT19 in laryngeal tumor tissue is associated with shorter overall survival time (Xu, Guo, and Zhang [15]). In this study, we observed that PCAT19 was lowly expressed in 11 types of cancers, especially in lung cancer tissues. Meanwhile, we found that PCAT19 level was appreciably downregulated in cancer tissues derived from LC patients, which was similar to the results of Acha-Sagredo et al. (Acha-Sagredo et al. [27]). Moreover, our survival analysis uncovered that the survival rate of LC patients with high expression of PCAT19 was much higher, indicating that the overall survival rate of LC patients was positively related to PCAT19 level. Furthermore, we analyzed the clinical features of LC patients with different expression levels of PCAT19 and discovered that tumor size and pathology were related to the expression of PCAT19.

Regulating gene expressions is effective in treating cancer (Belguise et al. [28], Sui et al. [29], Amirsaadat et al. [30]). At present, the roles of various genes in the regulation of LC progression have been increasingly investigated. For example, Cui et al. confirmed that SNHG1 was highly expressed in LC patients, and downregulation of SNHG1 could inhibit the growth of non-small-cell lung cancer (Cui et al. [31]). PCAT19 expression was downregulated in lung adenocarcinoma patient tissues, and overexpression of PCAT19 could signally hamper the proliferation, migration, and invasion of lung adenocarcinoma cells (Tang et al. [32]). In the current study, we obtained similar results, the PCAT19 overexpression vector and silencing vector were transfected into LC cells to investigate the effects on LC cells, and we observed that overexpression of PCAT19 repressed cell viability, reduced the cell colony number, and promoted apoptosis. Moreover, tumor formation experiments also verified that overexpression of PCAT19 suppressed tumor growth while promoting tumor cell apoptosis, indicating that regulation of PCAT19 expression could regulate the progression of LC.

miR-25-3p has been proven to be highly expressed in LC tissues (Giordano et al. [21]). Consistently, the current study also found the similar results by detecting the expression of miR-25-3p in LC tissues, but whether miR-25-3p was involved in the development of LC and whether it was related to PCAT19 have not been elucidated yet. In addition, a prior study pointed out that inhibition of BTG2 expression in breast cancer could indirectly activate AKT and ERK-MAPK signaling pathways, thereby mediating the downstream effects of miR-25-3p and controlling disease progression (Chen et al. [23]). On this basis, the current study found that MAP2K, an important factor in the MAPK cascade, had a binding site with miR-25-3p and that MAP2K4 level was apparently reduced in LC patients.

Studies have indicated that activation of the MAPK signaling pathway promotes the progression of gastric cancer cells (Mi et al. [33]), and increasing MAPK signaling in lung adenocarcinoma can promote rapid progression of adenomas to malignant adenocarcinoma (Cicchini et al. [34]). Therefore, we explored the effects of PCAT19 on the MAPK signaling pathway in LC cells and confirmed the targeted relationship between PCAT19 and miR-25-3p by *in vitro* experiments. ERK1/2, p38, and JNK pertain to the MAPK family (Gao, Shan, et al. [35], Bubici and Papa [36, 37]), and activation of ERK1/2 protein can promote the development of lung cancer in mice (Yamakawa et al. [38]), activation of p38 phosphorylation can enhance the production of tumor factors (Alam et al. [39]), and JNK can regulate a variety of cell biological functions. Additionally, the JNK protein expression has been reported to strengthen the activity of cancer cells (Wang, Ni, et al. [40]). In the current study, we found that overexpression of PCAT19 could downregulate the phosphorylation levels of MAPK signaling pathway-related proteins ERK1/2, p38, and JNK, thereby inhibiting the activation of the MAPK signaling pathway. However, PCAT19 silencing generated the opposite results. As evidenced by a prior study, the inhibition on the activation of the MAPK signaling pathway could repress the growth of H460 and H1299 LC cells (Liu et al. [41]). Furthermore, in this research, MAPK signaling pathway agonists were applied to treat the cells transfected with the PCAT19 overexpression vector, and the results signified that overexpression of PCAT19 hindered the progression of agonist-induced LC cells. Moreover, PCAT19 overexpression could hamper the viability and proliferation while promoting the apoptosis of LC cells through regulating the MAPK signaling pathway.

In previous reports, PCAT19 was proven to be able to facilitate tumor cell growth in non-small-cell lung cancer cells H1993 with the characteristic of lymphatic metastasis (Zhang et al. [42]) and in laryngeal cancer (Cossu et al. [43]). However, similar to TCGA data and the report of Acha-Sagredo et al. (Acha-Sagredo et al. [27]), data from this study suggested that PCAT19 may be a tumor suppressor in non-small-cell lung cancer cells A549 and lung squamous cells SK-MES-1. The discrepancy on the different functions of PCAT19 needs to be further deciphered in the future. In our study, the overexpressed PCAT19 markedly impacted the tumor cell behaviors.

## 5. Conclusions

In conclusion, the study reveals that upregulated PCAT19 suppresses the proliferation yet promotes the apoptosis of A549 and SK-MES-1 cells through modulating the miR-25-3p/MAP2K4 signaling axis.

## Figures and Tables

**Figure 1:** PCAT19 level was reduced in LC tissues. (a, b) GEPIA was used to predict PCAT19 expression in adenocarcinoma of lung and squamous cell carcinoma cells (^∗^*P* < 0.05). (c) Kaplan-Meier plotter was utilized to predict the relationship between PCAT19 and the survival of LC patients.Abbreviations: GEPIA: Gene Expression Profiling Interactive Analysis.

**Figure 2:** PCAT19 was lowly expressed in LC tissues and cells. (a) qRT-PCR was performed to quantify the expression of PCAT19 in the cancer tissues and ANT from 74 LC patients. (b) The expression of PCAT19 in 74 LC patients was detected by qRT-PCR. (c) The expression of PCAT19 in the human normal lung epithelial cell line (BEAS-2B) and LC cell line was determined by qRT-PCR (*n* = 3) (^∗∗∗^*P* < 0.001 vs. BEAS-2B). Abbreviations: ANT: paracancer tissues; LC: lung cancer; qRT-PCR: quantitative real-time polymerase chain reaction.

**Figure 3:** Upregulated PCAT19 inhibited LC cell proliferation while promoting LC cell apoptosis. (a, b) The expression of PCAT19 in A549 and SK-MES-1 cells transfected with the PCAT19 or siPCAT19 vector was detected by qRT-PCR. (c, d) The viability of A549 and SK-MES-1 cells transfected with the PCAT19 or siPCAT19 vector was detected by the MTT assay. (e, f) Colony formation assay was conducted to observe the growth of A549 and SK-MES-1 cells transfected with the PCAT19 and siPCAT19 vector. (g, h) Apoptosis of A549 and SK-MES-1 cells transfected with the PCAT19 or siPCAT19 vector was detected by flow cytometry. (i, j) Flow cytometry was used to detect the cycle of A549 and SK-MES-1 cells transfected with the PCAT19 or siPCAT19 vector. ^∗^*P* < 0.05, ^∗∗^*P* < 0.01, and ^∗∗∗∗^*P* < 0.001 vs. NC; ^#^*P* < 0.05, ^##^*P* < 0.01, and ^###^*P* < 0.001 vs. siNC. Abbreviations: LC: lung cancer; qRT-PCR: quantitative real-time polymerase chain reaction; MTT: methylthiazolyldiphenyl-tetrazolium bromide; NC: negative control.

**Figure 4:** Upregulated PCAT19 inhibited the growth of the tumor. (a–c) Tumor-bearing model was established in mice using A549 cells transfected with the NC and PCAT19 vector, and the tumor (a, b) volume (cm^3^) and (c) weight (g) were counted. (d) Ki-67 expression was detected by immunohistochemistry, and apoptosis was detected by the TUNEL assay. ^∗∗∗^*P* < 0.001 vs. NC. Abbreviations: TUNEL: terminal deoxynucleotidyl transferase (TdT) dUTP nick-end labeling assay; NC: negative control.

**Figure 5:** PCAT19 regulated the miR-25-3p/MAP2K4 signaling axis. (a) The expression of PCAT19 in the nucleus and cytoplasm of A549 cells was detected by qRT-PCR. (b) The expression of PCAT19 in the nucleus and cytoplasm of SK-MES-1 cells was quantified by qRT-PCR. (c) LncBase V.2 was used to predict the binding sites of PCAT19 and miR-25-3p. (d) PCAT19-WT or PCAT19-Mut was cotransfected with the miR-25-3p mimic into A549 cells, followed by the detection on the luciferase activity of the dual-luciferase reporter assay. (e) PCAT19-WT or PCAT19-Mut was cotransfected with the miR-25-3p mimic into SK-MES-1 cells, and then, the luciferase activity was determined by the dual-luciferase reporter assay. (f) TargetScan 7.2 was employed to predict the binding sites of MAP2K4 and miR-25-3p. (g) MAP2K4-WT or MAP2K4-Mut was cotransfected with the miR-25-3p mimic into A549 cells, and then, the dual-luciferase reporter assay was carried out. (h) MAP2K4-WT or MAP2K4-Mut was cotransfected with the miR-25-3p mimic into SK-MES-1 cells, subsequent to which the dual-luciferase reporter assay was applied to detect the luciferase activity. ^∗∗^*P* < 0.01, ^∗∗∗^*P* < 0.001 vs. nucleus; ^△△^*P* < 0.01, ^△△△^*P* < 0.001 vs. mimic+PCAT19-Mut or mimic+MAP2K4-Mut. Abbreviations: qRT-PCR: quantitative real-time polymerase chain reaction; WT: wild type; Mut: mutant.

**Figure 6:** Expression and correlation analysis of miR-25-3p and MAP2K4 in LC tissues. (a) The expression of miR-25-3p in cancer tissues and ANT of 74 LC patients was detected by qRT-PCR. (b) The expression of MAP2K4 in cancer tissues and ANT from 74 LC patients was measured by qPCR. (c–e) Spearman correlation analysis was performed to analyze the relationship between miR-25-3p and PCAT19 (c), miR-25-3p and MAP2K4 (d), and PCAT19 and MAP2K4 (e) in 74 LC patients. Abbreviations: ANT: paracancer tissues; LC: lung cancer; qRT-PCR: quantitative real-time polymerase chain reaction.

**Figure 7:** Upregulated PCAT19 inhibited the activation of the MAPK signaling pathway. (a, b) Western blotting was performed to detect the expressions of MAPK signaling pathway-associated proteins (p-ERK1/2, ERK1/2, p-p38, p-JNK, and JNK) in A549 cells. (c, d) Western blotting was conducted to determine the expressions of MAPK signaling pathway-associated proteins (p-ERK1/2, ERK1/2, p-p38, p-JNK, and JNK) in SK-MES-1 cells. (e) The ratios of MAPK signaling pathway-related proteins were determined in A549 cells. (f) The ratio of MAPK signaling pathway-related proteins was determined in SK-MES-1 cells. ^∗^*P* < 0.05, ^∗∗^*P* < 0.01, and ^∗∗∗^*P* < 0.001 vs. NC; ^##^*P* < 0.01, ^###^*P* < 0.001 vs. siNC. Abbreviations: JNK: c-Jun N-terminal kinase; MAPK: mitogen-activated protein kinase; qRT-PCR: quantitative real-time polymerase chain reaction; NC: negative control.

**Figure 8:** PCAT19 regulated LC cell growth and apoptosis by inhibiting the MAPK signaling pathway. (a, b) The viability of A549 and SK-MES-1 cells treated with Honokiol (10 *μ*M) of the ERK agonist and anisomycin (0.1 *μ*M) of the p38 and JNK agonist was detected by the MTT assay. (c, d) Colony formation assay was performed to observe the growth of A549 and SK-MES-1 cells treated with Honokiol (10 *μ*M) of the ERK agonist and anisomycin (0.1 *μ*M) of the p38 and JNK agonist. (e, f) Apoptosis of A549 and SK-MES-1 cells treated with Honokiol (10 *μ*M) of the ERK agonist and anisomycin (0.1 *μ*M) of the p38 and JNK agonist was detected by flow cytometry. ^∗^*P* < 0.05, ^∗∗∗^*P* < 0.001 vs. NC; ^^^*P* < 0.05, ^^^^*P* < 0.01, and ^^^^^*P* < 0.001 vs. Hon; ^##^*P* < 0.01, ^###^*P* < 0.001 vs. Ani. Abbreviations: ERK: extracellular regulated protein kinases; JNK: c-Jun N-terminal kinase; MAPK: mitogen-activated protein kinase; qRT-PCR: quantitative real-time polymerase chain reaction.

**Table 1:** Primers used in real-time PCR analysis.

Gene	Primer sequence	Species
PCAT19	Forward: 5′-CAGAACAGGATGGCAGAG-3′ Reverse: 5′-GGACTACTTGGATGGCTAAT-3′	Human
miR-25-3p	Forward: 5′-CATTGCACTTGTCTCGGTCTGA-3′ Reverse: 5′-GCTGTCAACGATACGCTACGTAACG-3′	Human
MAP2K4	Forward: 5′-GGCCAAAGTATAAAGAGCTTCTGA-3′ Reverse: 5′-CAGCGATATCAATCGACATACAT-3′	Human
U6	Forward: 5′-TGACTTCCAAGTACCATCGCCA-3′ Reverse: 5′-TTGTAGAGGTAGGTGTGCAGCAT-3′	Human
GAPDH	Forward: 5′-GGTGAAGGTCGGAGTCAACG-3′ Reverse: 5′-CAAAG TTGTCATGGATGTACC-3′	Human

Abbreviations: miRNA: microRNA.

**Table 2:** Relationship between PCAT19 expression level and clinical characteristics of lung cancer patients.

Variables	Patients (*n* = 74)	PCAT19 expression		*χ* ^2^	*P*
		High (*n* = 40)	Low (*n* = 34)		
Age (years)				0.031	0.859^∗^
<60	34	18 (52.94%)	16 (47.06%)		
≥60	40	22 (55.00%)	18 (45.00%)		
Gender				—	0.719^#^
Male	66	35 (58.33%)	31 (46.97%)		
Female	8	5 (62.50%)	3 (37.50%)		
Tumor size (cm)				7.551	0.006^∗^
<5	30	22 (73.33%)	8 (26.67%)		
≥5	44	18 (40.91%)	26 (59.09%)		
Pathology				8.867	0.012^∗^
LUAD	35	18 (51.43%)	17 (48.57%)		
LUSC	24	18 (75.00%)	6 (25.00%)		
Large-cell carcinoma	15	4 (26.67%)	11 (73.33%)		
Clinical stage				0.641	0.423^∗^
I-II	45	26 (57.78%)	19 (42.22%)		
III-IV	29	14 (48.28%)	15 (51.72%)		
Lymph node metastasis				0.804	0.370^∗^
Yes	35	17 (48.57%)	18 (51.43%)		
No	39	23 (58.97%)	16 (41.03%)		

^∗^ *P*: chi-squared test; ^#^*P*: Fisher exact test.

## Data Availability

The analyzed data sets generated during the study are available from the corresponding author on reasonable request.

## References

[1] Siegel R. L., Miller K. D., Fuchs H. E., Jemal A. (2021). Cancer statistics. *CA: a Cancer Journal for Clinicians*.

[2] Torre L. A., Bray F., Siegel R. L., Ferlay J., Lortet-Tieulent J., Jemal A. (2015). Global cancer statistics. *CA: a Cancer Journal for Clinicians*.

[3] Goubran H. A., Kotb R. R., Stakiw J., Emara M. E., Burnouf T. (2014). Regulation of tumor growth and metastasis: the role of tumor microenvironment. *Cancer Growth Metastasis*.

[4] Wangari-Talbot J., Hopper-Borge E. (2013). Drug resistance mechanisms in non-small cell lung carcinoma. *J Can Res Updates*.

[5] Baghdadi M., Endo H., Takano A. (2018). High co-expression of IL-34 and M-CSF correlates with tumor progression and poor survival in lung cancers. *Scientific Reports*.

[6] Avci N., Hayar M., Altmisdortoglu O. (2017). Smoking habits are an independent prognostic factor in patients with lung cancer. *The Clinical Respiratory Journal*.

[7] Granger C. L., Connolly B., Denehy L. (2017). Understanding factors influencing physical activity and exercise in lung cancer: a systematic review. *Support Care Cancer*.

[8] Dreher M., Kruger S., Schulze-Olden S. (2018). Sleep-disordered breathing in patients with newly diagnosed lung cancer. *BMC Pulmonary Medicine*.

[9] Zhao W., Huang C. C., Otterson G. A. (2012). Altered p16(INK4) and RB1 expressions are associated with poor prognosis in patients with nonsmall cell lung cancer. *Journal of Oncology*.

[10] Jiang S. S., Fang W. T., Hou Y. H. (2010). Upregulation of SOX9 in lung adenocarcinoma and its involvement in the regulation of cell growth and tumorigenicity. *Clinical Cancer Research*.

[11] Engreitz J. M., Haines J. E., Perez E. M. (2016). Local regulation of gene expression by lncRNA promoters, transcription and splicing. *Nature*.

[12] Liu Y., Zhao M. (2016). lnCaNet: pan-cancer co-expression network for human lncRNA and cancer genes. *Bioinformatics*.

[13] Wang S., Ren L., Shen G., Liu M., Luo J. (2020). The knockdown of MALAT1 inhibits the proliferation, invasion and migration of hemangioma endothelial cells by regulating MiR-206 / VEGFA axis. *Molecular and Cellular Probes*.

[14] Hua J. T., Ahmed M., Guo H. (2018). Risk SNP-mediated promoter-enhancer switching drives prostate cancer through lncRNA PCAT19. *Cell*.

[15] Xu S., Guo J., Zhang W. (2019). lncRNA PCAT19 promotes the proliferation of laryngocarcinoma cells via modulation of the miR-182/PDK4 axis. *Journal of Cellular Biochemistry*.

[16] Chen M. T., Lin H. S., Shen C. (2015). PU.1-regulated long noncoding RNA lnc-MC controls human monocyte/macrophage differentiation through interaction with microRNA 199a-5p. *Molecular and Cellular Biology*.

[17] Wang J., Jia Y., Zhao S. (2017). BIN1 reverses PD-L1-mediated immune escape by inactivating the c-MYC and EGFR/MAPK signaling pathways in non-small cell lung cancer. *Oncogene*.

[18] Yoon J. H., Abdelmohsen K., Gorospe M. (2014). Functional interactions among microRNAs and long noncoding RNAs. *Seminars in Cell & Developmental Biology*.

[19] Hao N. B., He Y. F., Li X. Q., Wang K., Wang R. L. (2017). The role of miRNA and lncRNA in gastric cancer. *Oncotarget*.

[20] He J. H., Han Z. P., Zou M. X. (2018). Analyzing the LncRNA, miRNA, and mRNA regulatory network in prostate cancer with bioinformatics software. *Journal of Computational Biology*.

[21] Giordano M., Boldrini L., Servadio A. (2018). Differential microRNA expression profiles between young and old lung adenocarcinoma patients. *American Journal of Translational Research*.

[22] Hu W. W., Chen P. C., Chen J. M. (2017). Periostin promotes epithelial-mesenchymal transition via the MAPK/miR-381 axis in lung cancer. *Oncotarget*.

[23] Chen H., Pan H., Qian Y., Zhou W., Liu X. (2018). MiR-25-3p promotes the proliferation of triple negative breast cancer by targeting BTG2. *Molecular Cancer*.

[24] Livak K. J., Schmittgen T. D. (2001). Analysis of relative gene expression data using real-time quantitative PCR and the 2^−*ΔΔ*C^_T_ method. *Methods*.

[25] Hu P., He J., Liu S., Wang M., Pan B., Zhang W. (2016). *β*2-Adrenergic receptor activation promotes the proliferation of A549 lung cancer cells via the ERK1/2/CREB pathway. *Oncology Reports*.

[26] Gao P., Xia J. H., Sipeky C. (2018). Biology and clinical implications of the 19q13 aggressive prostate cancer susceptibility locus. *Cell*.

[27] Acha-Sagredo A., Uko B., Pantazi P. (2020). Long non-coding RNA dysregulation is a frequent event in non-small cell lung carcinoma pathogenesis. *British Journal of Cancer*.

[28] Belguise K., Cherradi S., Sarr A. (2017). PKC*θ*-induced phosphorylations control the ability of Fra-1 to stimulate gene expression and cancer cell migration. *Cancer Letters*.

[29] Sui W., Shi Z., Xue W. (2017). Circular RNA and gene expression profiles in gastric cancer based on microarray chip technology. *Oncology Reports*.

[30] Amirsaadat S., Pilehvar-Soltanahmadi Y., Zarghami F., Alipour S., Ebrahimnezhad Z., Zarghami N. (2017). Silibinin-loaded magnetic nanoparticles inhibit hTERT gene expression and proliferation of lung cancer cells. *Artif Cells Nanomed Biotechnol*.

[31] Cui Y., Zhang F., Zhu C., Geng L., Tian T., Liu H. (2017). Upregulated lncRNA SNHG1 contributes to progression of non-small cell lung cancer through inhibition of miR-101-3p and activation of Wnt/*β*-catenin signaling pathway. *Oncotarget*.

[32] Tang X., Hua X., Peng X., Pei Y., Chen Z. (2021). Integrated dissection of lncRNA-miRNA-mRNA pairs and potential regulatory role of lncRNA PCAT19 in lung adenocarcinoma. *Frontiers in Genetics*.

[33] Mi Y., Zhang D., Jiang W. (2017). miR-181a-5p promotes the progression of gastric cancer via RASSF6-mediated MAPK signalling activation. *Cancer Letters*.

[34] Cicchini M., Buza E. L., Sagal K. M., Gudiel A. A., Durham A. C., Feldser D. M. (2017). Context-dependent effects of amplified MAPK signaling during lung adenocarcinoma initiation and progression. *Cell Reports*.

[35] Gao X., Shan W., Liu X., Zhang J., Zheng J., Yao H. (2018). JNK1/2 and ERK1/2 provides vital clues about tumor recurrence and survival in hepatocellular carcinoma patients. *Future Oncology*.

[36] Bubici C., Papa S. (2014). JNK signalling in cancer: in need of new, smarter therapeutic targets. *British Journal of Pharmacology*.

[37] Zhao R., Wang Y., Huang Y. (2017). Effects of fiber and probiotics on diarrhea associated with enteral nutrition in gastric cancer patients: a prospective randomized and controlled trial. *Medicine (Baltimore)*.

[38] Yamakawa K., Yokohira M., Nakano Y., Kishi S., Kanie S., Imaida K. (2016). Activation of MEK1/2-ERK1/2 signaling during NNK-induced lung carcinogenesis in female A/J mice. *Cancer Medicine*.

[39] Alam M. S., Gaida M. M., Bergmann F. (2015). Selective inhibition of the p38 alternative activation pathway in infiltrating T cells inhibits pancreatic cancer progression. *Nature Medicine*.

[40] Wang J., Ni W. H., Hu K. B. (2017). Targeting MUC1 and JNK by RNA interference and inhibitor inhibit the development of hepatocellular carcinoma. *Cancer Science*.

[41] Liu Z., Zheng Q., Chen W. (2017). Chemosensitizing effect of Paris saponin I on camptothecin and 10-hydroxycamptothecin in lung cancer cells via p38 MAPK, ERK, and Akt signaling pathways. *European Journal of Medicinal Chemistry*.

[42] Zhang X., Wang Q., Xu Y. (2019). lncRNA PCAT19 negatively regulates p53 in non-small cell lung cancer. *Oncology Letters*.

[43] Cossu A. M., Mosca L., Zappavigna S. (2019). Long non-coding RNAs as important biomarkers in laryngeal cancer and other head and neck tumours. *International Journal of Molecular Sciences*.

